# The effects of residual platelets in plasma on plasminogen activator inhibitor-1 and plasminogen activator inhibitor-1-related assays

**DOI:** 10.1371/journal.pone.0171271

**Published:** 2017-02-03

**Authors:** Marlien Pieters, Sunelle A. Barnard, Du Toit Loots, Dingeman C. Rijken

**Affiliations:** 1 Centre of Excellence for Nutrition, North-West University, Potchefstroom, North West province, South Africa; 2 Human Metabolomics, North-West University, Potchefstroom, North West province, South Africa; 3 Department of Hematology, Erasmus University Medical Center, Rotterdam, Netherlands; Institut d'Investigacions Biomediques de Barcelona, SPAIN

## Abstract

Due to controversial evidence in the literature pertaining to the activity of plasminogen activator inhibitor-1 in platelets, we examined the effects of residual platelets present in plasma (a potential pre-analytical variable) on various plasminogen activator inhibitor-1 and plasminogen activator inhibitor-1-related assays. Blood samples were collected from 151 individuals and centrifuged at 352 and 1500 *g* to obtain plasma with varying numbers of platelet. In a follow-up study, blood samples were collected from an additional 23 individuals, from whom platelet-poor (2000 *g*), platelet-containing (352 *g*) and platelet-rich plasma (200 *g*) were prepared and analysed as fresh-frozen and after five defrost-refreeze cycles (to determine the contribution of *in vitro* platelet degradation). Plasminogen activator inhibitor-1 activity, plasminogen activator inhibitor-1 antigen, tissue plasminogen activator/plasminogen activator inhibitor-1 complex, plasma clot lysis time, β-thromboglobulin and plasma platelet count were analysed. Platelet α-granule release (plasma β-thromboglobulin) showed a significant association with plasminogen activator inhibitor-1 antigen levels but weak associations with plasminogen activator inhibitor-1 activity and a functional marker of fibrinolysis, clot lysis time. Upon dividing the study population into quartiles based on β-thromboglobulin levels, plasminogen activator inhibitor-1 antigen increased significantly across the quartiles while plasminogen activator inhibitor-1 activity and clot lysis time tended to increase in the 4^th^ quartile only. In the follow-up study, plasma plasminogen activator inhibitor-1 antigen was also significantly influenced by platelet count in a concentration-dependent manner. Plasma plasminogen activator inhibitor-1 antigen levels increased further after complete platelet degradation. Residual platelets in plasma significantly influence plasma plasminogen activator inhibitor-1 antigen levels mainly through release of latent plasminogen activator inhibitor-1 with limited effects on plasminogen activator inhibitor-1 activity, tissue plasminogen activator/plasminogen activator inhibitor-1 complex or plasma clot lysis time. Platelets may however also have functional effects on plasma fibrinolytic potential in the presence of high platelet counts, such as in platelet-rich plasma.

## Introduction

Plasminogen activator inhibitor type-1 (PAI-1) is a serine protease inhibitor (serpin) [1, 2], which acts as a main inhibitor of fibrinolysis [3]. Elevated plasma PAI-1 levels have been associated with a risk for developing atherothrombosis [4–6] due to its antifibrinolytic properties, by reducing the clearance of fibrin in plaques [5], and also *via* its influence on cellular migration, matrix remodelling and activation of growth factors [7, 8]. Plasma PAI-1 exists either in an active or latent form, or in complex with tissue plasminogen activator (tPA) [9–11]. The active form of PAI-1 is unstable, with a half-life of approximately two to three hours, after which it will spontaneously convert to the inactive, latent form [9, 12]. PAI-1 is produced by various cells such as endothelial cells, hepatocytes, smooth muscle cells, adipocytes, and platelets [11, 13]. In platelets, PAI-1 is stored in the alpha granules and is released during platelet activation and aggregation [11, 14, 15].

Recently, there has been a debate about which form of PAI-1, or at least the relative proportion of each form, is released from the platelet alpha granules. It was traditionally believed that platelets store and release mainly latent PAI-1, since, only approximately 5–10% of PAI-1 antigen (PAI-1_ag_) was shown to be active in lysed platelet-rich plasma [16]. More recent studies however, suggest that platelets release a substantial amount of active PAI-1 [17–19]. This is due to the observed *de novo* synthesis of PAI-1 within platelets, which was indicated to remain active for over 24 hours [17]. Possible explanations for the contradictory evidence pertaining to platelet PAI-1 activity, could be due to the different approaches used in these experiments for preparing the platelet lysates (sonification and freezing and or thawing of the samples), which have been reported to influence the detection of PAI-1 [18]. Furthermore, the conversion of active PAI-1 to its latent state can be influenced by low temperatures, low pH and high salt concentrations [20]. It is however not clear as to how the PAI-1, released from the alpha granules of residual platelets in plasma, affects PAI-1 assays and PAI-1-related assays.

The overall aim of the study was therefore to investigate the effect of residual platelets in plasma, on various PAI-1 and PAI-1-related assays: PAI-1 activity (PAI-1_act_), PAI-1 antigen (PAI-1_ag_), and tPA/PAI-1 complex, as well as plasma fibrinolytic potential (a functional parameter of fibrinolysis, measured as plasma clot lysis time (CLT)). The study consisted of two sub-studies. In the first, varying centrifugation speeds (352 and 1500 *g*) were used to prepare platelet-containing plasma, from 151 participants in the Sympathetic activity and Ambulatory Blood Pressure in Africans (SABPA) study. The purpose of this sub-study was to determine the effect of residual platelets in plasma on various PAI-1 assay results, by relating these assays to a marker of platelet alpha granule release (beta thromboglobulin (βTG)). In this sub-study, absolute platelet counts were not measured, and additionally it was not possible to calculate to what degree plasma PAI-1 levels were influenced by *in vitro* platelet activation and or degradation. Additionally, Merolla *et al*. [21] found that different centrifugation speeds may result in different platelet populations, which could also have had an effect on our results. The purpose of the second study was, therefore, to determine the influence of actual platelet count on PAI-1_ag_, as the antigen assay was the assay found to be significantly influenced by plasma platelet content in the first sub-study. In the follow-up study, plasma was collected from 23 additional participants, and platelet count and size, in addition to βTG and PAI-1_ag_ concentrations, where determined from three different plasma preparations: platelet-poor plasma (PPP– 2000 *g*), platelet-containing plasma (352 *g*, in keeping with the first sub-study protocol) and platelet-rich plasma (PRP– 200 *g*). PPP was collected in citrate tubes, containing platelet stabilisers, in order to provide basal plasma PAI-1_ag_ levels without any of the influencing effects of *in vitro* platelet activation and/or degradation. Furthermore, the 352 *g* and 200 *g* citrated plasma samples were analysed not only as fresh-frozen, but also after five defrost-refreeze cycles, ensuring complete alpha granule release from the platelets, in order to determine the total platelet PAI-1_ag_ and βTG content.

## Materials and methods

### Study population and ethics–SABPA study

The Sympathetic activity and Ambulatory Blood Pressure in Africans (SABPA) study, was a cross-sectional study including 409 (202 men and 207 women) school teachers between the ages of 25–60 years, from the North West Province, South Africa. Of these participants 151 individuals were randomly selected for inclusion in the present study. All samples were analysed at the same time. Exclusion criteria were: elevated ear temperature, dependence or abuse of psychotropic substances, regular blood donors, and individuals vaccinated within the previous three months. The study complied with all applicable international regulations and the Helsinki declaration for investigation of human participants. The study was approved by the Health Research Ethics Committee (HREC) of the North-West University (NWU), Potchefstroom Campus (NWU-00016-10-A1).

### Study population and ethics–follow-up study

Twenty three individuals from the same socio-demographic profile as the SABPA study participants were recruited by means of a purposive sampling method from the Potchefstroom Campus of the NWU. The same inclusion and exclusion criteria as well as ethical principles were adhered to. The study was approved by the HREC of the NWU, Potchefstroom Campus (NWU-00016-10-A1). All samples were collected and analysed at the same time.

### Blood collection–SABPA study

Fasting blood samples with minimum stasis were collected from the antebrachial vein before 10:00 am. 3.2% Citrate samples were used for the analysis of PAI-1 (activity, antigen and tPA/PAI-1 complex), βTG and CLT. Samples were randomly divided into two groups. One half of the study population samples were centrifuged at 352 *g* and the other half at 1500 *g* for 15 minutes at 20°C to yield plasma containing a varying number of platelets. Aliquots were snap frozen on dry ice and stored at -82°C until analysis.

### Blood collection–follow-up study

Fasting blood samples with minimum stasis were collected from the antebrachial vein before 10:00 am. Blood was collected into two 3.2% citrated tubes and one CTAD tube (a citrate tube containing platelet stabilisers; theophylline, adenosine and dipyridamol). CTAD plasma was prepared by centrifuging the samples at 2000 *g* for 30 minutes at 20°C, to yield PPP with platelets protected from *in vitro* activation or degradation. Two types of citrate plasma were prepared by centrifuging one of the citrated tubes at 352 x *g* for 15 minutes at 20°C, to yield platelet-containing plasma, and the other tube at 200 x *g* for 10 minutes at 20°C, to yield PRP. These conditions were comparable to that of the SABPA study and also served the purpose to provide information on standard plasma type preparations–PPP and PRP. All samples were centrifuged within 20 min of collection.

Platelet count and size analyses were performed in fresh whole blood samples collected both in citrate and CTAD tubes, as well as in the different plasma preparations described above. The remaining plasma was then aliquoted, snap frozen on dry ice and stored at -82°C. The CTAD plasma samples and half of the aliquots of the two citrate plasma preparations, of each individual, were thawed once only, by placing these in a 37°C water bath for 10 minutes, immediately prior to PAI-1_ag_ and βTG analyses. The second half of the citrated plasma sample aliquots underwent five freeze-thaw cycles (x 5), once daily, prior to analysis, to ensure maximum platelet α-granule release. Fig 1 provides a schematic depiction of the study design.

**Fig 1:** Design of follow-up study.

### Biochemical analysis

PAI-1_act_ was measured using an indirect enzymatic method (Technozym PAI-1 Actibind, Technoclone, Vienna, Austria), and PAI-1_ag_, using a two-site enzyme-linked immunosorbent assay (ELISA) (TriniLIZE PAI-1_ag,_ TCoag, Bray Ireland). tPA/PAI-1 complex was analysed using a solid phase enzyme immunoassay, specific to PAI-1 complexed to tPA (Technoclone, Vienna, Austria). An ELISA assay was used to measure βTG levels (Asserachrom® βTG Diagnostica Stago, Asnières sur Seine, France). CLT was determined by studying the lysis of a tissue factor-induced plasma clot by exogenous tPA. Changes in turbidity during clot formation and lysis were monitored as described by Lisman *et al*. [22]. Tissue factor and tPA concentrations were slightly modified to obtain comparable CLTs of approximately 60 minutes. The modified concentrations were 17 mmol/L CaCl_2_, 60 ng/ml tPA (Actilyse, Boehringer Ingelheim, Ingelheim, Germany) and 10 μmol/L phospholipids vesicles (Rossix, Mölndal, Sweden). Tissue factor was diluted 3000 times (Dade Innovin, Siemens Healthcare Diagnostics Inc., Marburg, Germany). CLT was defined as the time from the midpoint, from clear to maximum turbidity (representative of the clot formation), to the midpoint in the transition from maximum turbidity to the final baseline turbidity (representative of the lysis of the clot) [22]. Platelet count and mean platelet volume were determined with a Coulter AcT 5-part differential (5 diff) autoloader haematology analyser (Beckman Coulter, Fullerton, CA, USA).

### Statistical analysis

The data was analysed with the computer software package Statistica (Statsoft Inc., Tulsa Oklahoma, USA). A p-value of 0.05 or less was regarded as statistically significant. Descriptive data is presented as median (25^th^; 75^th^ percentiles) as most of the variables were not normally distributed. Kruskal-Wallis analysis of variance (ANOVA) with multiple comparisons of mean post-hoc tests were used to compare differences in the PAI-1 and CLT assays, between population sub-groups divided into quartiles of βTG levels. Correlations between variables were determined both with Spearman Rank order and Pearson (for log transformed data) correlation tests. Only the Spearman data is reported, as both correlation tests provided similar results. Significant differences between correlation coefficients obtained were also calculated. For the follow-up study, Wilcoxon-Matched pairs tests were used to determine significant differences between plasma prepared at 200 and 352 *g* and also between fresh-frozen and 5 times defrosted-refrozen samples.

## Results

### SABPA study

The study population included 151 participants, with a mean age of 45.7 (±8.75) years and a BMI of 26.9 (±2.29). When comparing the samples prepared at the two different centrifugation speeds, the 352 *g* group had significantly higher βTG (3263 vs 355 IU/mL; p < 0.0001) and PAI-1_ag_ (33.8 vs 20.8 ng/mL; p < 0.0001) levels, compared to the 1500 *g* group, with borderline significantly higher PAI-1_act_ (2.95 vs 1.91 U/mL; p = 0.03) and longer CLT (78.2 vs 74.4 min; p = 0.04). No difference in tPA/PAI-1 complex (p = 0.09) was observed (Table 1).

**Table 1:** Comparison of βTG, PAI-1 assays and CLT according to centrifugation speed in SABPA study.

Variable	352 *g* (n = 75)	1500 *g* (n = 75)	
	Median (25^th^; 75^th^ percentiles)	Median (25^th^; 75^th^ percentiles)	p-value(Mann-Whitney)
βTG (IU/mL)	3263 (2009; 4394)	355 (218; 584)	<0.0001
PAI-1 _ag_ (ng/mL)	33.8 (28.4; 42.4)	20.8 (16.7; 25.8)	<0.0001
PAI-1_act_ (U/mL)	2.95 (0.69; 8.72)	1.91 (0.25; 4.68)	0.03
tPA/PAI complex (ng/mL)	8.78 (6.59; 11.7)	7.90 (6.01; 10.2)	0.09
CLT (min)	78.2 (69.7; 86.4)	74.4 (69.7; 79.8)	0.04

βTG—beta thromboglobulin; CLT—clot lysis time; PAI-1 –plasminogen activator inhibitor-1 PAI-1_act_−PAI-1 activity; PAI-1 _ag_−PAI-1 antigen; tPA/PAI complex—tissue plasminogen activator/PAI-1 complex.

When dividing the study population into quartiles according to plasma βTG levels (Table 2), PAI-1_ag_ increased consistently across the βTG quartiles. PAI-1_act_ showed a significant increase in the highest βTG quartile only, with CLT tending to be longer, without reaching significance. No difference was observed in tPA/PAI-1 complex across the βTG quartiles. βTG was furthermore correlated with PAI-1_ag_ (r = 0.66; p<0.0001), demonstrating statistically weaker correlations with PAI-1_act_ (r = 0.22; p = 0.008); tPA/PAI-1 complex (r = 0.12; p = 0.13) and CLT (r = 0.20; p = 0.02) (Table 3). CLT showed the strongest correlation with PAI-1_act_ (r = 0.74; p<0.0001).

**Table 2:** PAI-1_act_, PAI-1_ag_, tPA/PAI-1 complex and CLT according to βTG quartiles in SABPA study group.

Variable	SAPBA study group								
	βTG 1^st^ Quartile(≤341 IU/mL)		βTG 2^nd^ Quartile(341 IU/mL—817 IU/mL)		βTG 3^rd^ Quartile(817 IU/mL—3263 IU/mL)		βTG 4^th^ Quartile(>3263 IU/mL)		ANOVA p-value
	n	Median (25; 75% percentile)	n	Median (25; 75% percentile)	n	Median (25; 75% percentile)	n	Median (25; 75% percentile)	
PAI-1_ag_ (ng/L)	37	20.4 (16.0; 25.8) *	38	21.5 (17.0; 26.7) *	37	29.6 (25.1; 39.7) ^#^	37	40.7 (31.0; 42.9) ^#^	<0.0001
PAI-1_act_ (U/mL)	34	2.56 (0.31; 4.89)	37	1.89 (0.20; 3.77) *	37	1.37 (0.41; 6.70)	36	5.65 (1.28; 10.3) ^#^	0.03
tPA/PAI-1 complex (ng/mL)	35	8.00 (6.36; 10.2)	37	7.55 (5.26; 10.1)	37	8.65 (6.28; 11.7)	38	9.06 (7.32; 11.3)	0.1
CLT (min)	34	75.4 (69.7; 79.5)	37	73.9 (69.7; 78.6)	36	76.6 (67.7; 84.1)	35	81.5 (71.6; 96.0)	0.06

ANOVA, analysis of co-variance; βTG, beta thromboglobulin; CLT, clot lysis time; PAI-1, plasminogen activator inhibitor-1; PAI-1_act_, PAI-1 activity; PAI-1 _ag_, PAI-1 antigen; tPA/PAI-complex, tissue plasminogen activator/PAI-1 complex

* ^#^ Medians with different symbols differ significantly.

**Table 3:** Spearman rank order correlations between βTG, PAI-1 assays and CLT in SABPA study group.

Variables	βTG r (p-value)	PAI-1 _ag_ r (p-value)	PAI-1_act_r (p-value)	tPA/PAI-1complexr (p-value)
PAI-1 _ag_ (ng/mL)	0.66 (<0.0001)	-	-	-
PAI-1_act_ (U/mL)	0.22 (0.008) *	0.43 (<0.0001)	-	-
tPA/PAI-1 complex (ng/mL)	0.12 (0.13) *	0.30 (0.0002)	0.64 (<0.0001)	-
CLT (min)	0.20 (0.02) *	0.41 (<0.0001)	0.74 (<0.0001)	0.50 (<0.0001)

βTG, beta thromboglobulin; CLT, clot lysis time; PAI-1, plasminogen activator inhibitor-1; PAI-1_act_; PAI-1 activity; PAI-1 _ag_, PAI-1 antigen; tPA/PAI-complex, tissue plasminogen activator/PAI-1 complex.

* Significantly weaker correlation with βTG than the correlation of PAI-1_ag_ with βTG.

### Follow-up study

Table 4 presents the descriptive statistics of the follow-up study group. Platelet counts in the citrated and CTAD whole blood were similar. The platelet count of the CTAD samples centrifuged at 2000 *g* was 1.00 (1.00–2.00) x 10^3^/μL, confirming that it was indeed platelet poor (<10 x 10^3^/μL). The platelet counts of the 352 *g* and 200 *g* plasma were 323 (257–440) x 10^3^/μL and 523 (389–674) x 10^3^/μL respectively. The 352 *g* plasma had a significantly lower mean platelet volume (7.00 [6.65–7.60] fL) than the 200 *g* plasma (7.80 [7.00–8.30] fL), which in turn had a similar mean platelet volume than that of the whole blood. βTG levels increased 60 fold and 150 fold in the 352 *g* and 200 *g* plasma respectively, compared to the PPP, while PAI-1_ag_ levels increased 15 and 22 fold respectively. In both the 352 *g* and 200 *g* plasma, the βTG levels of the samples that underwent 5 freeze-thaw cycles, prior to analyses, were significantly lower than that of the samples that were defrosted once only, prior to analysis, possibly due to instability of βTG (5% and 3% respectively), while PAI-1_ag_ levels showed significant increases of 26% and 27% respectively.

**Table 4:** Descriptive statistics of the follow-up study group.

Variable	Study population (n = 23)
	Median (25^th^; 75^th^ percentiles)
Gender: men / women (n)	12 / 11
Ethnicity: black / white (n)	11 / 12
Age (years)	36 (29; 42)
SBP (mm Hg)	120 (110; 130)
DBP (mm Hg)	80 (70; 80)
BMI (kg/m^2^)	26.4 (22.0; 28.4)
CTAD whole blood platelet count (x10^3^/μL)	239 (195; 248)
Citrate whole blood platelet count (x10^3^/μL)	234 (194; 257)
CTAD plasma 2000 *g* platelet count (x10^3^/μL)	1.00 (1.00; 2.00)
Citrate plasma 352 *g* platelet count (x10^3^/μL)	323 (257; 440)
Citrate plasma 200 *g* platelet count (x10^3^/μL)	523 (389; 674)
Whole blood CTAD MPV (fL)	7.80 (7.40; 8.40)
Whole blood Citrate MPV (fL)	7.80 (7.20: 8.30)
MPV (fL) 352 *g* plasma	7.00 (6.65; 7.60)^%^
MPV (fL) 200 *g* plasma	7.80 (7.00; 8.30)^%^
βTG (IU/mL) CTAD 2000 *g* plasma	120 (92; 156)
βTG (IU/mL) 352 *g* x 1 plasma	7269 (6218; 8902)^#^
βTG (IU mL) 352 *g* x 5 plasma	6890 (5770; 7985)^#^
βTG (IU/mL) 200 *g* x 1 plasma	17683 (14703; 19089)^^^
βTG (IU/mL) 200 *g* x 5 plasma	17182 (14322; 18393)^^^
PAI-1_ag_ (ng/mL) CTAD 2000 *g* plasma	5.16 (3.80; 11.5)
PAI-1_ag_ (ng/mL) 352 *g* x 1 plasma	76.7 (64.1; 86.0)^$^
PAI-1_ag_ (ng/mL) 352 *g* x 5 plasma	96.9 (74.7; 117)^$^
PAI-1_ag_ (ng/mL) 200 *g* x 1 plasma	114.2 (90.6; 155)^&^
PAI-1_ag_ (ng/mL) 200 *g* x 5 plasma	145 (115; 191)^&^

BMI, body mass index; βTG, beta thromboglobulin; CTAD, citrate-theophylline, adenosine, dipyridamol; DBP, diastolic blood pressure; *g*, gravitational acceleration; PAI-1, plasminogen activator inhibitor-1; PAI-1_ag_, PAI-1 antigen; SBP, systolic blood pressure; MPV, mean platelet volume

^# ^ $ & % @ **^ Median with the same symbol differ significantly between the 1x and 5 x frozen and defrosted samples.

When combining the different types of plasma, βTG had a highly significant correlation with platelet count (r = 0.91, p<0.0001). When investigating the different types of plasma separately, βTG levels correlated well with platelet count in the 352 *g* (r = 0.60, p = 0.002) and 200 *g* (r = 0.70, p = 0.0002) plasma samples, with a smaller and non-significant correlation (r = 0.40, p = 0.06) in the PPP (Table 5). For all the types of plasma combined, PAI-1_ag_ and platelet count were highly correlated (r = 0.91, p<0.0001). Compared with βTG, PAI-1_ag_ showed even stronger statistical correlations with platelet count in the 352 *g* (r = 0.85, p<0.0001) and 200 *g* (r = 0.81, p<0.0001) plasma. None of the plasma preparations’ βTG levels correlated with whole blood platelet count, while the correlation of PAI-1_ag_ of the 200 *g* plasma with whole blood platelet count, reached borderline significance (r = 0.4, p = 0.06). Furthermore, βTG and PAI-1_ag_ correlated significantly when combining the different types of plasma (r = 0.86, p<0.0001), however, correlated negatively in PPP (r = -0.61, p = 0.002), with significant positive correlations in the 352 *g* (r = 0.55, p = 0.006) and 200 *g* (r = 0.74, p<0.0001) plasma separately (Table 6).

**Table 5:** Spearman rank order correlations of βTG and PAI-1_ag_ with whole blood, CTAD and citrate plasma platelet count of the follow-up study.

Variable	Platelet count x10^3^/μl (n = 23)						
	CTAD whole blood r (p-value)		CTAD plasma (2000 *g*) r (p-value)		Citrate whole blood r (p-value)	Citrate plasma (352 *g*)r (p-value)	Citrate plasma (200 *g*) r (p-value)
βTG (IU/mL) CTAD 2000 *g* plasma		-0.14 (0.5)	0.40 (0.06)	-		-	-
βTG (IU/mL) 352 *g* x 1 plasma		-	-	0.12 (0.6)		0.6 (0.002)	-
βTG (IU/mL) 200 *g* x 1 plasma		-	-	0.20 (0.3)		-	0.70 (0.0002)
PAI-1_ag_ (ng/mL) CTAD 2000 *g* plasma		0.04 (0.9)	-0.36 (0.09)	-		-	-
PAI-1_ag_ (ng/mL) 352 *g* x 1 plasma		-	-	0.34 (0.1)		0.85 (<0.0001)	-
PAI-1_ag_ (ng/mL) 200 *g* x 1 plasma		-	-	0.40 (0.06)		-	0.81 (<0.0001)

βTG, beta thromboglobulin; CTAD, citrate-theophylline, adenosine, dipyridamol; *g*, gravitational acceleration; PAI-1, plasminogen activator inhibitor-1; PAI-1 _ag_, PAI-1 antigen.

**Table 6:** Spearman rank order correlations between βTG and PAI-1_ag_ in the respective plasma preparations of the follow-up study.

Variables	βTG—PAI-1_ag_r (p-value)
CTAD plasma 2000 *g*	-0.61 (0.002)
Citrate plasma 352 *g* x 1	0.55 (0.006)
Citrate plasma 200 *g* x 1	0.74 (<0.0001)

βTG, beta thromboglobulin; CTAD, citrate-theophylline, adenosine, dipyridamol; *g*, gravitational acceleration; PAI-1, plasminogen activator inhibitor-1; PAI-1 _ag_, PAI-1 antigen.

## Discussion

This study investigated the effect of residual platelets present in plasma, on plasma PAI-1 and PAI-1-related assay results. The presence of platelets in plasma significantly influenced plasma PAI-1_ag_ levels in a concentration dependent manner, likely due to an increase in mainly plasma latent PAI-1. Only in the presence of large amounts of platelets such as in PRP, functional effects in terms of plasma fibrinolytic potential are seen, suggesting the presence of a comparatively lower concentration of active PAI-1 in platelets. It was furthermore demonstrated that platelets present in plasma, do not initially release all of their PAI-1 content and that further release of PAI-1 can occur upon further / complete *in vitro* platelet degradation.

### SABPA study

The SABPA study data indicated that βTG levels had a significantly stronger association with PAI-1_ag_ levels than any of the other PAI-1 variables or CLT. When dividing the study population into βTG quartiles, PAI-1_act_ and CLT increased in the highest βTG quartile only, suggesting that there may be a small amount of active PAI-1 present in platelets. In agreement with this, Serizawa *et al*. [23] found longer CLT in PRP than PPP which was ascribed to the presence of active PAI-1 in platelets. Since PAI-1_ag_ is composed of latent PAI-1, active PAI-1 and PAI-1 in complex with tPA, the data suggests that platelet alpha granule release largely contributes to increased plasma PAI-1_ag_, by increasing latent PAI-1. It was unfortunately not possible to measure plasma latent PAI-1 levels directly, as no such commercial assay is currently available. Latent PAI-1 is unable to inhibit tPA; therefore, the presence of latent PAI-1 in plasma may lead to a falsely assumed increased fibrinolytic inhibitory capacity. The lack of increase in CLT across the βTG quartiles, (apart from the highest quartile) confirms this. These results are also in agreement with a study by Juhan-Vague *et al*. [24] who found PAI-1, released from platelets, *in vitro*, to be mainly in the inactive form. Combined, this data suggests that platelets likely contain both latent and active PAI-1, but that a high plasma platelet content (such as in PRP) is required before the active PAI-1 present in platelets has functional effects on plasma fibrinolytic potential.

### Follow-up study

Data from the follow-up study, clearly demonstrated the significant effects of platelets present in plasma, on plasma PAI-1_ag_ levels. Platelet count and βTG and PAI-1_ag_ levels were highly correlated in the different plasma preparations containing platelets (352 *g* and 200 *g*), with no significant associations in the PPP. PAI-1_ag_ levels in PRP already tended to correlate with whole blood platelet count. PAI-1_ag_ levels, were furthermore, up to 22 fold higher in PRP when compared to basal levels in PPP (which was exempted from the possible influence of residual platelet content or *in vitro* platelet α-granule release), highlighting the magnitude of the effect of platelets on plasma PAI-1_ag_ levels, compared to other sources of PAI-1 (endothelial cells, hepatocytes, smooth muscle cells and adipocytes) [11, 13]. The additional 1.3 fold increase in plasma PAI-1_ag,_ subsequent to maximal degradation (5 x freeze-that cycles), suggests that *in vitro* platelet degradation can contribute to a further increase in plasma PAI-1_ag_ levels, confirming the necessity of the use of the correct plasma preparation protocols to standardise platelet count and to ensure the preparation of platelet-poor plasma (<10 x 10^3^/μL). Differences in platelet size were also detected when comparing the 352 *g* and the 200 *g* plasma, indicating the presence of different platelet populations in the samples centrifuged at different speeds. Since platelets with larger sizes are known to be more metabolically active than smaller platelets [25], platelet size, in addition to platelet count, most likely influence the relationship between platelets present in plasma and PAI-1_ag_ levels.

Although βTG is extensively used as a marker of platelet alpha granule release, it does have limitations. The sensitivity of βTG as a marker of platelet activation and alpha granule release can be influenced by various factors; including the choice of anticoagulant, and sample handling and preparation procedures [26, 27]. The significant correlation between platelet count and βTG (r = 0.91, p<0.0001) does however support its use as a proxy marker for the number of platelets in plasma in our study populations. While PAI-1 activity may be influenced by freeze-thaw cycles, we opted to work with frozen samples as this type of sample is most often used in studies and therefore relevant to a larger audience. It should be noted that since all samples were frozen at least once, possible effects of freezing on platelet function cannot be excluded. All plasma preparations were however treated similarly making comparison between the different preparations possible. Although samples were not specifically treated to prevent possible *in vitro* conversion of active to latent PAI-1, samples were processed within 20 minutes after collection and snap frozen to limit *in vitro* conversion.

The results from the present study indicate that the content of the alpha granules released from platelets in plasma, significantly influences plasma PAI-1_ag_ levels, with limited effects on PAI-1_act_, tPA/PAI-1 complex or fibrinolysis rate (measured as CLT). This effect on PAI-1_ag_ is thought to be largely due to an increased release of latent PAI-1 from platelets which is unable to bind tPA and inhibit fibrinolysis. Due to the potential contribution of latent PAI-1 to PAI-1_ag_ levels, PAI-1_act_ may be the more clinically useful assay to determine the fibrinolytic inhibitor capacity of plasma. In plasma with a high platelet count, such as PRP, the component of platelet PAI-1 that is active, may, however have functional effects by decreasing plasma fibrinolytic potential. These results suggest that PAI-1_ag_ is more sensitive to the presence of platelets in plasma, than other PAI-1 assays (PAI-1_act_ and tPA/PAI-1 complex) or CLT but that these assays may also be influenced by platelets when present in high numbers such as in PRP.

## Supporting information

S1 Data SABPA study. (XLSX)

S2 Data Follow-up study. (XLSX)

## Abbreviations

βTG: beta thromboglobulin
CLT: clot lysis time
CTAD: citrate-theophylline, adenosine, dipyridamole
ELISA: enzyme-linked immunosorbent assay
HREC: Health Research Ethics Committee
MPV: mean platelet volume
NWU: North-West University
PAI-1: plasminogen activator inhibitor-1
PAI-1_act_: PAI-1 activity
PAI-1_ag_: PAI-1 antigen
PPP: platelet-poor plasma
PRP: platelet-rich plasma
tPA/PAI-1 complex: tissue plasminogen activator/PAI-1 complex
SABPA: Sympathetic activity and Ambulatory Blood Pressure in Africans
